# Rescue of MHC-1 Antigen Processing Machinery by Down-Regulation in Expression of IGF-1 in Human Glioblastoma Cells

**DOI:** 10.1371/journal.pone.0058428

**Published:** 2013-03-20

**Authors:** Yuexin Pan, Jerzy Trojan, Yajun Guo, Donald D. Anthony

**Affiliations:** 1 Division of General Medical Sciences, School of Medicine, Case Western Reserve University, Cleveland, Ohio, United States of America; 2 Department of Medicine, University Hospitals of Cleveland, Cleveland, Ohio, United States of America; 3 INSERM U542 and U602, Paul-Brousse Hospital, Paris XI University, Villejuif, France; 4 International Joint Cancer Institute, Second Military Medical University, Shanghai, China; University of Navarra, Spain

## Abstract

Escape from immune recognition has been hypothesized to be a factor in carcinogenesis. It may be mediated for many cancers through down-regulation in the MHC class 1 antigen processing and presentation pathway. TAP-1, TAP-2, tightly linked to LMP-2 and LMP-7 are multiple components of the endogenous, antigen presentation pathway machinery. We addressed the question of alterations in this pathway in human Glioblastoma (HGB) and of its relationship to modulation in expression of IGF-1 that is highly expressed in this cancer. Deficiencies in expression of TAP-1 were demonstrated by RT-PCR and/or by immuno-flow cytometry in the HGB cell line T98G obtained from ATCC, and in 3 of 4 human cell lines established from patients with Glioblastoma Multiforme. Deficiencies in expression of TAP-2 were observed in 3 of 4, deficiencies in expression of LMP-2 in 4 of 4 and deficiencies in LMP-7 in 3 of 4 HGB cell lines examined by RT-PCR and Western blot. Following down-regulation of IGF-1 by transfection with the pAnti IGF-1 vector that expresses IGF-1 RNA in antisense orientation, or by the exogenous addition of IGF-1 receptor monoclonal antibody to cell culture media, the deficiencies in components of the MHC-1 antigen presentation pathway were up-regulated and/or rescued in all HGB cell lines tested. Moreover, this up-regulation in expression was aborted by addition of 100 ng/ml of IGF-1 to the culture media. Unlike in the case of IFN-γ, the restoration of TAP-1 and LMP-2 by down-regulation of IGF-1 in Glioblastoma cells was not correlated to the tyrosine phosphorylation of STAT 1. In summary, the simultaneous reversion in expression of the multiple constituents of MHC-1 antigen processing path and up-regulation in expression of MHC-1 occurring with down-regulation in IGF-1 may have a role in reinforcement of immunity against tumor antigen(s) in some animal cancers and in humans with Glioblastoma Multiforme.

## Introduction

Major histocompatibility complex (MHC) genes in humans are referred to as human leukocyte antigen (HLA) genes. The HLA locus spans approximately four megabases on chromosome 6P21.3. Its gene products are predominately associated with the immune system. HLA-1 and II molecules are membrane-bound glyco-proteins, which have key roles in the presentation of antigens to T-lymphocytes [1], [2]. HLA-1 molecules are ubiquitously expressed in accordance with their essential functions in mediating immune responses against endogenously derived virus and tumor cell antigens [3]. Endogenous antigen peptides are generally produced in the cytosol by large multicatalytic proteolytic molecules named proteasomes (LMPs). LMP-2, LMP-7 and LMP-10 subunits of the proteasomes are inducible by interferon-gama (IFN-γ) [4], [5]. The 8–9 amino acids antigen peptides produced by this reaction are then translocated to the endoplasmic reticulum (ER) by transporters associated with antigen processing (TAP-1 and TAP-2) [6], [7]. Assembly with HLA class 1 heavy chain and the β_2_-microglobulin light chain occurs here [8]. The HLA class 1 peptide complex is then transported to the cell surface to be presented to cytotoxic T lymphocytes (CTL). This antigen-processing machinery and HLA-1 restricted antigen-presentation pathway is believed to have a role in the activation of CTL mediated immunogenicity [9]. Importantly, this machinery and the MHC-1 restricted antigen presentation pathway are down-regulated in many different cancer tissues and cancer cell lines [10]–[14]. This has led to the hypothesis that the defective pathway may have a significant role in loss of immuno-surveillance and possibly in causation of cancer.

We previously showed, in several different animal cancer models (rat C6 glioma [15], murine teratocarcinoma [16], transgenic spontaneous hepatoma [17], commentary rat/LFCI2A-hepatocarcinoma [18]), and, in human glioblastoma cell lines [19], an up-regulation in expression of MHC class 1 following down-regulation in cellular IGF-1 by transfection with the pAnti IGF-1 (an IGF-1 antisense RNA expression vector) [19]–[21]. We show in this paper, the association between down–regulation in expression of IGF-1 and enhancement in the cell surface expression of HLA class 1 molecules in human Glioblastoma cells and Glioblastoma cell lines. Along with this, we show a concomitant increase in mRNA expression for TAP-1, TAP-2, LMP-2 and LMP-7 components of the endogenous antigen presentation pathway. Increase in the TAP-1 peptide was demonstrated, and, increase and/or rescue in the expression of TAP-2, LMP-2 and LMP-7 peptides were demonstrated when down-regulation of IGF-1 by IGF-1 antisense RNA or when blockade of the IGF-1 receptor (IGF-1R) by its monoclonal antibody occurred. We conclude that loss and/or down-regulation in expression of the endogenous antigen processing pathway machinery in human Glioblastoma (HGB) and HGB cell lines can be modulated and rescued by down-regulation of IGF-1 expression in HGB cells.

## Materials and Methods

### Ethical Considerations

Human experiments were done in accordance with the Declaration of Helsinki (1964). The experiments were conducted with the understanding and informed consent of the human subjects. The Institutional Review Board of University Hospitals of Cleveland has approved these experiments.

### Cell Lines and Cell Culture

The human Glioblastoma cell line T98G was obtained from the American Type Culture Collection (ATCC, Rockville, MD). Primary human Glioblastoma cell lines were obtained from 16 patients with diagnosis of human Glioblastoma multiforme as determined by histo-pathology in accordance with the World Health Organization system of classification. Primary human Glioblastoma cell cultures were derived according to techniques previously described [22]. Cells were grown in supplemented Dulbecco's Modified Eagle's medium (DMEM) containing 4.5 g/l Glucose, 4 mM L-Glutamine (Biowhittaker) to which was added 1×non-essential amino acids solution (MEM) (GIBCO/BRL, Carlsbad, CA), 1 mM sodium pyruvate (GIBCO/BRL), 5 μg/ml human transferrin (GIBCO/BRL), 3.46 ng/ml sodium selenite (GIBCO/BRL) and 500 ng/ml insulin (SIGMA, St. Louis, MO). The complete medium was adjusted to a final concentration of 10% fetal bovine serum (FBS) (Biowhittaker, Walkersville, MD). Cultures were maintained in a humidified atmosphere of 5% CO_2_ and 95% air at 37°C.

### pAnti IGF-1 Plasmid

The *E. coli* bacterial strain DH5α bearing the IGF-1 antisense RNA vector, pAnti-IGF-1, was kindly provided by Dr. J. Ilan (Case Western Reserve University, Cleveland, Ohio, USA). This expression vector includes the Epstein-Barr virus origin of replication and the gene encoding nuclear antigen 1, which together drive extra-chromosomal replication. The construct shown in **Fig 1A** is as previously described [22]. The vector replicates episomally within human cells providing a copy number up to 100 per cell [23]. Vector is isolated and purified using a Plasmid Maxi Kit (QIAGEN, Valencia, CA) according to manufacturer's instructions. A control plasmid, pAnti IGF-2 has the same construction map accept the 1 kb of IGF-2 cDNA, in antisense orientation, replaced the IGF-1 antisense sequence. This was also previously described by us [16].

**Figure 1:** Transfection of HGB cells with the vector pAnti IGF-1. **A,** Physical map of pAnti IGF-1. MT-1: metallothionein - 1 promotor; IGF-1 3′-5′: human IGF-1 DNA sequence in antisense orientation; SV40 poly A: SV40 poly A termination sequence; Ori: origin of replication; Hyg R: hygromycin resistance gene; Amp R: Ampicillin resistance gene; EBNA-1: Epstein Barr Virus (EBV) encoded nuclear antigen 1; EBV ori-P: EBV origin of replication. **B,** Expression of IGF-1 cDNA in transfected HGB cells. Primer pairs for RT-PCR used to detect and amplify antisense IGF-1 cDNA are as designated in methods. This set of primers gives rise to a 424 bp cDNA band containing exons 1, 2, 3 and 5 of the IGF-1 molecule in antisense orientation. Lane 1 shows the molecular weight markers of ØX174 DNA cut by HaeIII. Lanes 2, 3 and 4 demonstrate the 424 bp band, and a 327 bp β-actin band (internal control). Lane 5 shows a negative clone, which did not express IGF-I antisense cDNA. Lane 6 depicts a negative control in which all constituents of the reaction were present but not the DNA template. **C,** Detection of IGF-1 antisense RNA transcripts in HGB cells by Northern blot analysis. 30ug of total RNA from non-Transfected and transfected clones of HGB cells were applied to 1.0% formaldehyde agarose gel. ^32^P-labeled IGF-I cDNA was used as probe. Lanes 1, 3, 4, 5, 6, 8, 9 and 10 demonstrate the dominant 1 kb IGF-1 antisense RNA band from each of 8 separately transfected clones. Lanes 2, 7 and 11 represent RNA of non-transfected clones. **Fig 1** **C** represents result for one set of the experiments; **Fig 1** **D** represents the semi-quantitative densitometry analysis for **C** as determined by the NIH image J program.

### Transfection of Human Glioblastoma Cells

The ATCC human glioblastoma (HGB) cell line T98G and cell lines established in our laboratory from primary cultures of HGB patients were transfected with pAnti IGF-1 as previously described using the lipofectin reagent kit available from GIBCO/BRL [22]. Isolated foci (clones) of transfected cells were obtained using cloning cylinders. Separated clones were transferred to six-well plates, expanded and transferred to 60 mm or larger culture dishes as appropriate. The populations of cells were then further expanded under growth conditions that included the selective pressure of hygromycin B. Cell passages used to reach the point at which transfection could be done were 1 – 2 [22]. To complete transfection to point of a stably transfected cell line required an additional 3 – 4 cell passages.

### Immunofluorescent Flow Cytometry

Immunofluorescent staining for HLA Class 1 and B-7.1 antigens was performed by modification of standard techniques at 4°C in a 96 well micro-titer plate [22]. HGB cells were first trypsinized and washed×3 with phosphate buffered saline (PBS) as previously described. Cells (2.5 – 5.0×10^5^) in 150 μl PBS were loaded into each well of a 96 well plate and centrifuged 800 g×5 min at 4°C. Supernatants were aspirated and primary antibody was added at a dilution of 1∶50 at 4°C for 30 min. Cells were then washed×3 with 150 μl of PBS as previously described [22]. Secondary antibody binding was performed using fluorescein isothiocyanate (FITC) conjugated goat anti-mouse IgG (Kirkegaard & Perry Lab, KPL, Gaithersburg, MA) at a dilution of 1∶200 in absence of light. Surface antigen B-7.1 was detected, using mouse anti-human B-7.1 monoclonal antibody conjugated with R-phycoerythrin (R-PE) (Ancell, Bayport, MN), by direct staining technique in the absence of light. To detect intracellular IGF-1 and TAP-1, trypsinized and PBS washed cells were pretreated with 2% paraformaldehyde at 25°C ×5 minutes and permeabilized with 0.1% Triton x-100 at 25°C for 1 min. Cells were treated with primary antibody, mouse anti-human IGF-1 (Upstate Biotechnology, Waltham, MA) or mouse anti-human TAP-1 antibody (a gift from Dr. Robert Tampe, Philipps-University of Marburg, Germany), and, then stained with secondary antibody (FITC conjugated goat anti-mouse IgG) and analyzed by flow cytometry (Becton Dickinson, Franklin Lakes, NJ) on the day of staining. Histogram analysis was performed using LYSYS II software.

For immuno-cytochemistry and flow cytometry studies, non -transfected or transfected cells were incubated×18–20 hrs in supplemented DMEM (with no added FBS) in presence or absence of 50 uM ZnSO_4_. Incubations were done to complete induction and expression of IGF-1 antisense RNA and the down-regulation of IGF-1 prior to cell staining procedures.

### PCR and RT-PCR

Cell lysates were prepared for polymerase chain reaction (PCR) by addition of cells in 100 ul aliquots of PCR buffer (50 mM KCL, 10 mM Tri-HCL pH 8.3, 2.5 mM MgCL_2_) containing the 0.45% non-ionic detergent NP40, 0.45% Tween-20 and 100 µg/ml proteinase K, to each well of a 48 well-plate. Following incubation×1 hr at 55°C, temperature was increased to 95°C ×10 min to inactivate proteinase K. Detection of IGF-1 antisense cDNA by PCR was carried out in a Thermal Cycler 480 (Perkin Elmer) programmed for 30 cycles of 60/45/90 sec at 94/56/72°C respectively, using *Taq* polymerase. Reverse transcription PCR (RT-PCR), for detection of IGF-1 antisense RNA and TAP-1, TAP-2, LMP-2, and, LMP-7 mRNA, was performed using Trizol reagent (GIBCO/BRL) in the presence of RNase inhibitor (RNasin). Briefly, HGB cells cultured in 100 mm dishes were washed with PBS×1, PBS was aspirated and 2 ml of Trizol reagent was added to each dish. The mixtures were then incubated at room temperature×5 min. 0.4 ml of chloroform was added and the homogenates were formed with gentle shaking. After incubation×2 min at room temperature, mixtures were centrifuged at 1,500 rpm×7min at 4°C to separate phases. The upper aqueous phase was transferred to a fresh tube, mixed with an equal volume of isopropyl alcohol and then incubated at room temperature×10 min. Total RNA precipitates were obtained by centrifugation at 12,000 g×15 min at 4°C in a microfuge. Pellets were washed×1 in 75% ethanol, air-dried and re-suspended in DEPC (diethylpyrocarbonate)-treated water. DNase digestion was then done in 50 ul aliquots of total RNA as previously described [22]. After incubation at 37°C ×I hr, 100ul of Trizol reagent+20 ul of chloroform were added and reactions were continued at 25°C ×5 min. The mixtures were then centrifuged at 12,000 g×15 min at 4°C in a micro-centrifuge. The upper phases were separated and precipitated with an equal volume of isopropyl alcohol. The pellets were washed with 75% alcohol and air-dried×5 min. Reverse transcription was done as follows: 16ul (2 uM) of the DNAse treated total RNA was combined with 5ul (1.5 uM) random primer (GIBCO/BRL), 10 ul of 5×RT-buffer and 6.5ul of DEPC-treated water; and, the mixture was then incubated at 70°C ×5 min. After chilling on ice, 5ul of M-MLV (Moloney Murine Leukemia Virus) reverse transcriptase (200 u/ul), 5ul of 0.1 M DDT, 1ul of 4×dNTP and 1.5ul of 40u/ul RNasin were added. The reaction was then incubated at 42°C ×50 min, and terminated at 99°C ×5 min. PCR was carried out combining 2.5 ul of the cDNA solution, 2.5 ul of 10×PCR buffer, 0.75ul of 50 mM MgCL_2_, 1.25 ul of dNTP mix (4 mM each), 1.0 ul of the forward and reverse primer pair (50 ng), 0.5 µl of the β-actin primer pair (50 ng), 0.25 ul of Taq polymerase (0.5u) and 15.5 ul of water. PCR was done in a Perkin Elmer thermal cycler 480 as previously described. The sequences of primer pairs used for amplification of cDNA are shown in **Table 1**.

**Table 1:** Primer pairs used for RT-PCR.

Product	5′ Sequence 3′	Function	Length of cDNA
ANTISENSE IGF1	GAAGATGCACACCATGTCCT	Forward	424 bp
	TCACTCTTCACTCCTCAGGAG	Reverse	
TAP-1	GGGCTGTAAGCAGTGGGAACC	Forward	197 bp
	CAAGGCCCTCCAAGTGTAAGGG	Reverse	
TAP-2	CACGGCTGAGCTCGGATACCAC	Forward	428 bp
	CGACTCAGCATCAGCATCTGC	Reverse	
LMP-2	GGGATAGAACTGGAGGAACC	Forward	312 bp
	AGATGACACCCCCGCTTGAG	Reverse	
LMP-7	GAACACTTATGCCTACGGGGTC	Forward	174 bp
	TTTCTACTTTCACCCAACCATC	Reverse	

### Western Immunobloting

HGB cells grown to 90% confluence were incubated in fresh serum-free, supplemented DMEM containing 50 µM ZnSO4×18–20 hrs. Cells were washed ×1with cold 1×DPBS, then solubilized in 0.5 ml of cold lysis buffer cocktail containing protease inhibitors (complete mini) (Roche, Indianapolis, IN) at 4°C. Cell lysates were sonicated×10–15 sec to shear DNA and reduce viscosity of samples. Protein concentration was determined for samples, using the DC protein assay kit (Bio-Rad laboratories, Hercules, CA). 50 µg of each sample was heated to 95–100°C ×5 min, cooled in ice and centrifuged at 12,000 g×5 min. Supernatants were maintained at room temperature, then loaded on SDS-PAGE gel and electrophoresis was carried out at 125 V for 1 hr. The separated proteins were electro-transferred to PVDF membrane (Immobilon^™^– P membrane) (Millipore, Bedford, MA) at 30 V overnight or at 120 V for 1 hr at 4°C. Non-specific protein binding was blocked by incubation in TBS-T (20 mM Tris/HCL, PH 7.6, 137 mM NaCL, 0.1% Tween 20) containing 5% non-fat milk for 1 hr at room temperature. Immuno-detection was performed using primary mouse anti-human TAP-1 monoclonal antibody (a gift from Dr. Robert Tampe, Philipps-University of Marburg, Germany) and secondary rabbit anti-mouse IgG antibody conjugated with horseradish peroxidase (HRP) (Cell Signaling Technology, Beverly, MA). LumiGLO chemiluminesence was used as the detection system. Blots were stripped with Western-Re-Probe (Gene Technology, Inc, St. Louis, MO) and probed with primary mouse anti-human actin (Ab-1) monoclonal antibody (IgM) and secondary goat anti-mouse IgM antibody conjugated with HRP (Oncogene Research Products, San Diego, CA).

### Quantification and Statistical Analysis

Quantification by densitometry for images from RT-PCR was performed with an Epson Scanner densitometer. The relative optical densities were measured by sampling 5×5 pixels. The density for each sample band was determined relative to the corresponding band of actin, with subtraction of the background density for a similar-sized area in a control zone of the image section. The quantity of each protein band in the Western blot was determined using the NIH IJ (image J) densitometry program. Statistical analysis was performed using SDA WINKS Software (Cedar Hill, Texas). All values are expressed as means (+/-SEM) for similar sized samples from two - three independent experiments. The One-way ANOVA/t-test analysis of variance was performed to assess significance. P Values<0.05 were considered statistically significant.

## Results

### Molecular Characterization and Down-regulation of IGF-I in pAnti-IGF-I Transfected HGB Cell Lines

Human Glioblastoma (HGB) cell lines, obtained from primary cultures of six patients with histo-pathologically diagnosed Glioblastoma, each demonstrated glial fibrillary acidic protein (GFAP) and IGF-1 positivities by indirect immuno-cytochemical staining technique using mouse anti-human IGF-1 monoclonal antibody. IGF-1 positive cells were characterized by yellow-brown staining in peri-nuclear cytoplasm. The HGB cell line T98G, obtained from ATCC, demonstrated similar staining. In contrast, pAnti-IGF-1 transfected HGB cells stained negatively [22]. **Fig 1** **A** shows a map of the 10.8 kb pAnti-IGF-1 vector. This plasmid expresses 1 kb of IGF-1 RNA in antisense orientation. The suppression of endogenous cellular IGF-1 RNA transcripts by IGF-1 antisense RNA in tumor cells was previously described [16], [24]. Data in **Fig1 B** show that IGF-I cDNA product from pAnti-IGF-1 vector in transfected cells was present in antisense orientation. In 3 of 4 separate clones tested using a primer pair that bridges IGF-I cDNA from exons 1 to 5, the PCR product was a 424 bp fragment characteristic of the IGF-I cDNA, which contains exons 1, 2, 3 and 5 but not exon 4 (lanes 2, 3, 4). This band was not appreciable in the RNA obtained from non-transfected cells (lane 5). The number of copies of vector in transfected cells was estimated by restriction enzyme analysis and Southern blot. The 10.8 kb DNA fragment characteristic of extra-chromosomal pAnti-IGF-I vector averaged 4 –10 copies per Human Glioblastoma transfected cell (data not shown). The expression of the 1 kb IGF-I antisense RNA in separately transfected cell clones is demonstrated by Northern blot in **Fig 1** **C** (lanes I, 3, 4, 5, 6, 8, 9, 10). The degree of expression varies greatly among different transfected cell clones. Lanes 2, 7 and 11 demonstrate that there was no hybridization of the IGF-I cDNA probe to RNA of non-transfected cell clones. **Fig 1** **D** represents a bar graph of quantitated intensities from bands shown in **Fig 1** **C**. Analysis by flow cytometry showing down-regulation of IGF-I in pAnti-IGF-I transfected, compared to non-transfected and mock transfected HG-2 cells is depicted in **Fig 2** **A**. Among the different HGB cell lines tested, IGF-I levels, as determined by specific fluorescence, were decreased variably by 28 to 93% in transfected (TX) relative to corresponding non-transfected (NT) clones (**Fig 2** **B**).

**Figure 2:** Down-regulation in expression of IGF-1 in pAnti IGF-1 transfected HGB cell lines. A, Demonstration of intracellular IGF-1 levels in the HG-2 cell line by Flowcytometry. Isotype control (non-transfected Cells+mouse IgG FITC); Non-transfected (non-transfected cells+mouse anti-human IGF-1 mAb+goat antimouse IgG FITC); Transfected (transfected cells+mouse antihuman IGF-1 mAb+goat antimouse IgG FITC); Mock transfected (cells transfected with vector minus antisense IGF-1 cDNA+mouse antihuman IGF-1 mAb+goat antimouse IgG FITC). **B,** Bar graph comparison of IGF-1 expression in transfected and corresponding parental, non-tranfected HGB Cell Lines. Cell lines were established from discarded tumor tissue of Glioblastoma patients. The experiment design was as depicted in legend **A** of this Fig. % IGF-1 content = %Fs (specific fluorescence) = [Target (Fluorescence mean value) – Control (Fluorescence mean value)]/Target (Fluorescence mean value)×100%. NT = non-transfected, TX = pAnti-IGF-1 transfected. The experiments of **Fig 2B** were done×3. The paired t-test was used to determine P values. The statistical procedures were performed on the average difference for each cell line before (NT) and after (TX) transfection. The calculated t and associated p-values are given. Grouped comparisons between TX and NT cell lines for IGF-1 from summarized data by two-way ANOVA were statistically significant at p<0.001 (5 cases) or p <0.05 (3 cases).

### Major Histocompatibility Complex (HLA-1) and Co-stimulatory B-7.1 in pAnti-IGF-1 Transfected HGB Cell Lines

Expression of HLA -1 in transfected compared to non-transfected clones of 6 separate HGB cell lines and the ATCC cell line T98G were analyzed by immunofluorescent flow cytometry. Similar comparisons were obtained for the expression of the B-7.1 co-stimulatory molecule in 4 of the 6 HGB cell lines. Each of the pAnti-IGF-1 transfected HGB cell lines tested was down-regulated in IGF-1 content. IGF-1 was also down-regulated by 90% in the transfected T98G cell line (data not shown). The results for up-regulation of HLA-1 and B-7.1 are summarized in **Table 2**. Parental T98G cells and 6 HGB cell lines expressed low levels of HLA-1 molecules on cell surfaces. Following transfection with pAnti-IGF-1, transfectants of the T98G cells and each of the 6 HGB cell lines tested showed a greater than 45% increase, with a range of increase up to seven fold in expression of HLA-1 (p< 0.05). Analysis by Flow cytometry demonstrating relatively significant increase in expression of HLA-1 in transfected, when compared to non-transfected and mock transfected, T98G cells is depicted in **Fig 3** **A** and **B** (P<0.05). Also depicted in **Figure 3** is transfection with the vector pAnti-IGF-2. These data showed no significant differences from the non-transfected or mock transfected controls (**Fig 3** **C**). Two HGB cell lines, HG-2 and HG-3, showed a 16 fold and 5 fold increase, respectively, in expression of the B-7.1 (**Table 2**). However, the increments of change in 2 of the 4 HGB cell lines tested (HG-4 and HG-25) were not sufficient to give statistically significant results.

**Figure 3:** Comparison of HLA-1 cell surface antigens in pAnti IGF-1 transfected, mock transfected, pAnti IGF-2 transfected and non-transfected T98G cells. A, Histogram of fluorescence intensity from isotype control (non-transfected cells+mouse IgG FITC); NT (non-transfected cells+mouse anti-human HLA-1 mAb+goat anti-mouse IgG FITC); Mock TX (cells transfected with vector devoid of anti IGF-1 cDNA+mouse anti-human HLA-1 mAb+goat anti-mouse IgG FITC); pAnti IGF-2 TX (cell transfected with vector expressing IGF-2 RNA in antisense orientation+mouse anti-human HLA-1 mAb+goat anti-mouse IgG FITC); and, pAnti IGF-1 TX (cells transfected with vector pAnti IGF-1+mouse anti-human HLA-1 mAb+goat anti-mouse IgG FITC). B, Specific fluorescence showing differential expression of HLA-1 from pAnti IGF-1 transfected cells when compared to parental non-transfected cells and other controls (P <0.05). C, Group ANOVA comparison was done by boxplot with Newman-Keuls graphical representation for comparison in expression of HLA-1 in the experimental groups. The data in Fig 3 B was repeated×3.

**Table 2:** Comparison in expression of HLA-1 and B-7.1 for pAnti IGF-1 transfected and non-transfected HGB cell lines by flow cytometry.

Cell line		HLA-1%Fs	B-7.1%Fs
HG-1	Control	22.1	ND
	TX	32.1	
	% change	+45.0	
	SD	1.13	
	P value	P = 0.019	
HG-2	Control	21.7	3.9
	TX	63.3	66.6
	% change	+191.7	+1607.0
	SD	2.65	10.15
	P value	P = 0.001	P = 0.008
HG-3	Control	12.5	7.5
	TX	36.3	45.1
	% change	+190.4	+501.3
	SD	4.41	1.65
	P value	P = 0.007	P = 0.001
HG-4	Control	17.8	44.9
	TX	35.6	45.8
	% change	+100.0	+2.0
	SD	1.58	1.56
	P value	P = 0.025	P = 0.766
HG-9	Control	6.3	ND
	TX	54.4	
	% change	+763.5	
	SD	4.13	
	P Value	P = 0.001	
HG-25	Control	11.9	27.6
	TX	50.9	33.0
	% change	+327.7	+19.6
	SD	4.13	1.50
	P value	P = 0.001	P = 0.07
T98G	Control	20.8	ND
	TX	35.9	
	% change	+72.6	
	SD	3.14	
	P value	P = 0.001	

Fs: Specific fluorescence. Fs defined as total mean fluorescence of sample (Ft) minus that of the background fluorescence (Fb) divided by Ft, i.e. %Fs = (Ft-Fb)/Ft×100.

Control: cells not transfected with vector pAnti IGF-1.

TX: cells transfected with vector pAnti IGF-1.

SD: standard deviation.

P value: Grouped comparison of TX vs. NT (control) by two-way ANOVA at p<0.05 is statistically significant.

### Enhanced Expression of TAP-1, TAP-2, LMP-2 and LMP-7 mRNA

Analysis by semi-quantitative RT-PCR demonstrated a relative decrease or absence in transcription of antigen processing products in 4 different parental, non-transfected, compared to corresponding transfected HGB cell lines. The data are shown in **Fig 4** **A** and **B** Lanes 1, 2, 3, 4 compared to lanes 5, 6, 7, 8 for TAP-1 and TAP-2 gene expression respectively, and, in **Fig 4** **C** and **D** lanes 1, 2, 3, 4 compared to lanes 5, 6, 7, 8 for LMP-7 and LMP-2 gene expression respectively. Following transfection, increases in the expression of TAP-1 mRNA, LMP-2 and LMP-7 mRNA for HG-3 were relatively less than in the cases of other transfected cell lines, accept in the case of TAP-2 mRNA (see lanes 6 of respective photographs). In two of the non-transfected cell lines, HG-5 and HG-9, TAP-2 mRNA expression was modest (lanes 3 and 4 of **Fig 4** **B**). However, its expression in transfected HG-5 and HG-9 cells in comparison to the corresponding non-transfected cells was substantially increased (lanes 7 and 8 of **Fig 4** **B**). Using the Epson perfection photo scanner, the optical intensities for **Fig A, B, C** and **D** are shown by the bar graphs of **Fig E, F, G, H**, respectively. The panels of each bar graph represent intensity in expression of the component molecule for each cell line as depicted. The intensity was calculated against intensity of the internal control, β-actin. Also subtracted was background in each of the respective sites. According to these measurements as shown in **Figs E**, **F**, **G** and **H**, following transfection the expression in TAP-1 was increased in HG-2, HG-5 and HG-9 (p<0.05); expression in TAP-2 was increased in HG-2 (p<0.001) and HG-3 (p<0.05); expression in LMP-7 was enhanced in HG-2 (p<0.001), HG-5 and HG-9 (p<0.05); and, expression in LMP-2 was up-regulated in HG-2 (p<0.001), HG-5 and HG-9 (p<0,05). These increments of increase are significant.

**Figure 4:** Comparison in expression of TAP and LMP transcripts in pAnti IGF-1 transfected (TX) and non-transfected (NT) HGB cell lines. RNA was prepared from cell lines established from four different patients. Following incubation of cells in the presence of 50 µM ZnSO_4_ for 18–20 hrs, agarose gel eletrophoresis and ethidium bromide staining were used to characterize products of RT-PCR for A, TAP-1; B, TAP-2; C, LMP-7; and D, LMP-2. Primer pairs for β-actin were included in each experiment as internal control. Expected sizes of RT-PCR products were: TAP-1, 197 bp; TAP-2, 428 bp; LMP-7, 174 bp; LMP-2, 312 bp; β-actin, 289 bp except in experiments concerning expression of LMP-2 in which the primer pair for the 618 bp fragment was used. Molecular weight markers are multiples of 50 bp from 50 to 800. Please note that Fig 4 A – D represent the results for one set of three similar RT-PCR experiments; E – H represent the results for the three sets of data analyzed together using the Epson Scan program for densitometry. Each TX cell line was compared to the respective NT cell line. Significance ** p<0.05, *** p<0.001.

### Up-regulation of TAP-1 and LMP-7 Peptides, and, Rescued Expression of TAP-2, LMP-2 Peptides and the B-7.1 Molecule

Down-regulation of IGF-1 or the IGF-1/IGF-1R signaling pathway by transfection with the pAnti- IGF-1 vector or by the exogenous addition of IGF-1R monoclonal antibody (mAb) to culture medium of HGB cell lines resulted in enhanced and/or rescued expression in antigen processing machinery components by Western Immuno-blotting analysis. **Fig 5** **A** demonstrates two transfectants, one from T98G and one from HG-2. Both showed a 70 kd band characteristic of the TAP-1 peptide. The corresponding non-transfected (NT) T98G and HG-2 cell lines did not show this band. Data are consistent with results from the RT-PCR experiments of **Fig 4**. **Fig 5** **B** demonstrates that three cell lines (T98G, HG-2 and HG-9) cultured in medium plus 10 ug/ml of IGF-1R monoclonal antibody were up-regulated in expression of TAP-1 and LMP-7, and that rescue in the expression of TAP-2 and LMP-2 occurred when compared to these cell lines cultured in medium minus the IGF-1R mAb. In **Fig 5** **B** row 5, the up-regulated expression of the co-stimulatory 60 kd B-7.1 molecule is also shown in these cell lines following blockade of the IGF-1 receptor by its monoclonal antibody. **Fig 5** **C** demonstrates the densities of the protein bands in Western blot of **Fig 5** **B**, and in an additional set of data from repeated experiments**,** as determined by the NIH image J program. It was shown that each of the components of the antigen processing machinery tested in these three HGB cell lines were significantly up-regulated following addition of the IGF-1R mAb to culture media (P<0.05).

**Figure 5:** Comparison in expression of TAP, LMP and B-7.1 peptides in parental and pAnti IGF-1 transfected and/or IGF-1R monoclonal antibody (mAb) treated HGB cell lines. A, Regulation of TAP-1 peptide in T98G and HG-2 TX cells was determined by Western Blot. Cell lysate was prepared from cells of TX and corresponding NT cell lines pretreated as described in Fig 4 and then subjected to SDS-PAGE and electronically blotted to nitrocellulose membrane. TAP-1 peptide on the membrane was probed by anti-human TAP-1 monoclonal Ab+anti-mouse IgG HRP-linked Ab; and, signal was detected by LumiGLO reagent. Lanes 1, 2 are NT cells from the T98G and HG-2 cell lines respectively. Lane 3, 4 are TX cells from clone b and c of the T98G cell line; Lane 5, 6 are TX cells from clone 5 and 11 of the HG-2 cell line. Re-probed membrane with anti-actin Ab demonstrates presence of the 42 kd actin. Up-regulation in expression of the 70 kd TAP-1 in the two pAnti IGF-1 transfected cell clones were demonstrated in this experiment. B, Up-regulation in TAP-1 and LMP-7 peptides, and, rescue in expression of TAP-2 and LMP-2 peptides following the exogenous addition of 10ug/ml IGF-1R mAb into cell culture medium for 48 hours were demonstrated by Western Blot. The lysates of wild type and IGF-1R antibody treated cells were prepared as described in A. Lanes 1, 2 and 3 represent T98G, HG-2 and HG-9 cell lines cultured in medium with no IGF-1R mAb added, while lanes 4, 5 and 6 are the corresponding respective cell lines cultured in medium with addition of exogenous IGF-1R mAb (10ug/ml), respectively. Rows 1, 2, 3 and 4 represent TAP-1, TAP-2, LMP-2 and LMP-7, respectively. Row 5 demonstrates the rescue in expression of the B-7.1 peptide in IGF-1R mAb treated T98G, HG-2 and HG-9 cell lines when compared to the wild types of the corresponding non-treated cells. The 42 kd band of actin is also shown as an internal control for the quantity of samples loaded. B represents the results from one set of the experiments, that were repeated×2; C, The densitometry analysis for the two sets of similar experiments was obtained by the NIH image J program. The differences in results between the groups with and without IGF-1R mAb in culture media were significant at p<0.05 or p<0.001.

### Specificity for Enhanced Expression of the TAP-1 peptide in pAnti-IGF-1 Transfected HGB Cell Lines

Quantitative assessment of intracellular TAP-1 peptide in HGB cell lines was demonstrated by immunofluorescent flow cytometry using mouse anti-human TAP-1 mAb as primary antibody (kindly provided by Dr. Robert Tampe, Philipp-University, Marburg, Germany). Enhancement of intracellular TAP-1 level was demonstrated in 8 pAnti-IGF-1 transfected T98G, 2 pAnti-IGF-1 transfected HG-2 and 1 pAnti-IGF-1 transfected HG-3 clones when compared to the respective non-transfected cell clones. The variation in degree of enhancement in transfected compared to corresponding non-transfected cell lines is shown in **Fig 6** **A**. The increase in each cell line is statistically significant at the p<0.05. **Fig 6** **B** and **C** demonstrate the relative specificity for enhancement of TAP-1 in pAnti IGF-1 transfected cells. For this experiment, the established ATCC T98G cell line was used. The data show a five fold increase in TAP-1 in pAnti IGF-1 transfected, IGF-1 down-regulated cells (8 clones), when compared to non-transfected cells (4 clones); a greater than 3 – 4 fold increase when compared to pEMT (vector containing no IGF-1 antisense sequence) transfected cells (4 clones), or to pAnti IGF-2 transfected cells (4 clones) (P<0.001). The degree of significance is shown in the **Fig 6** **C** box plot as determined by one-way ANOVA analysis. The results of the analysis showed that the group 4, T98G cells transfected with pAnti IGF-1, is significantly different from the other treatments (P<0.001); the differences between groups 1 (NT), 2 (EMP), and 3 (pAnti IGF-2) are not significant (P = 0.46).

**Figure 6:** Variability and specificity in expression of TAP-1 in HGB cell lines. A, Variability of TAP-1 levels in pAnti IGF-1 transfected and non-transfected HGB cell lines. Different clones of transfected (TX) and corresponding non-transfected (NT) HGB cell lines, eight from T98G (circles), two from HG-2 (rectangles) and one from HG-3 (triangle), were examined by flow cytometry for the expression of TAP-1. Expression of TAP-1 in TX and NT cell clones were determined using mouse anti-human TAP-1 monoclonal antibody (courtesy of Dr.Robert Tampe) as described in methods. The up-regulated expression of TAP-1 in TX compared to NT clones was significant at the P< 0.05. **B,** Relative specificity in up-regulation of TAP-1 in pAnti IGF-1 transfected HGB cells. T98G cells were transfected with the vector containing antisense IGF-1 cDNA (TX pAnti IGF-1), with vector containing antisense IGF-2 cDNA (TX pAnti IGF-2), or, with vector containing no antisense sequence (TX pEMT). Transfected cells were comparatively examined by flow cytometry relative to non-transfected T98G cells (NT) for content of TAP-1. The antibody used and flow cytometry analysis were as described in **A** of this Fig and methods. This experiment was repeated×3. **C,** TAP-1 expression in comparison of treatments was tested by t-test/ANOVA using Winks SDA software. Boxplot illustrates the comparison in specific fluorescence value among the experimental groups, P<0.001. Represented below the boxplot is the graphical description of Newman-Keuls multiple comparisons.

### Enhanced Expression of TAP-1 Peptide in pAnti IGF-1 Transfected HGB Cells was Down-regulated by Exogenous Addition of IGF-1

To detect whether the enhanced expression of TAP-1 peptide can be suppressed by IGF-1, the pAnti-IGF-1 transfected T98G and HG-2 cells were first cultured in serum- free medium in the presence of ZnSO4 (50uM) ×8 hours (Zn2+ binds to metal responsive element of metallothionein-1 promoter in the pAnti IGF-1 vector. This activates transcription of down-stream IGF-1 antisense cDNA). The cell culture was then incubated with addition of IGF-1 (100 ng/ml) overnight. The cell lysates of IGF-1 treated and transfected HGB cells were subjected to analysis by Western blot. The down-regulation in expression of TAP-1, after addition of IGF-1, in tested TX cell lines is shown in **Fig 7** **A**. The data showed that exogenous IGF-1 can reverse the up-regulation of TAP-1 that occurs with antisense IGF-1 transfection. The kinetics of decrease in expression of TAP-1 in pAnti IGF-1 transfected T98G cells by addition of IGF-1 (100 ng/ml) is shown in **Fig 7** **B, C**. In this case, the expression of TAP-1 was abolished after 60 minutes of treatment with IGF-1. The data therefore also demonstrate that IGF-1 may be involved in regulation of the TAP-1 gene expression.

**Figure 7:** Effect of exogenous IGF-1 on expression of TAP-1, pStat1(Tyr701) and pStat3(Tyr705). A, Expression of TAP-1 peptide in T98G cells was down-regulated by addition of IGF-1 to culture medium. TX cells were incubated in absence of serum and in the presence of 50 μM ZnSO_4_ and IGF-1 (100 ng/ml) over-night. Lanes 1 and 2 are NT cells from the T98G and HG-2 cell lines respectively. Lane 3 and lane 4 are T98G TX (clone b) and HG-2 TX (clone 5), respectively, into which IGF-1 was added overnight. Lanes 5 and 6 are as in lanes 3 and 4 except without added IGF-1. **B.** The expression of TAP-1 was examined as a function of time following addition of IGF-1 (100 ng/ml) in TX T98G cells in absence of serum and in the presence of Zn2+. Cells were treated with exogenous IGF-1 for the time periods as depicted. The cell lysates were prepared and subjected to Western Blot analysis as described in methods. The primary antibodies to TAP-1, pStat1 (Tyr701), pStat3 (Tyr705) and Stat3 were also obtained as described. The 70 kd TAP-1, 91 kd pStat1, and 86 kd pStat3 and 86 kd Stat3 peptides produced during the time course were identified by monoclonal antibody used and molecular weights. The data represent one of three sets of similar experimental results. **C,** Data from **Fig 7** **B** and similar results from two repeat experiments were used for this bar graph. The densitometry quantification was done using the NIH image J program as described in methods.

### Down-regulation in Expression of TAP-1 in pAnti IGF-1 Transfected HGB Cells by Exogenous Addition of IGF-1 Occurs with Inhibition of Phosphorylated STAT3(Tyr 705) and in Absence of Phosphorylated STAT1(Tyr 701)

In order to determine whether Stat signaling is involved in the IGF-1 regulated expression of the TAP-1 gene, the pAnti IGF-1 transfected T98G and/or HG-2 cells were treated with addition of IGF-1 (100 ng/ml) in absence of serum and with ZnSO_4_ (50uM) added to culture medium. During different time intervals of treatment, cells were collected and cell lysates were obtained as described in methods and analyzed by Western blot using the antibodies (Cell Signaling Technology Inc.) specific for phosphorylated Stat1(Tyr 701) or phosphorylated Stat3(Tyr 705). The expression of pStat1 in T98G NT (data not shown) and T98G TX cells was not detected; and it was also not detected after the exogenous addition of IGF-1 (**Fig 7** **B, C**). In contrast, pStat3 was expressed in both T98G NT (data not shown) and T98G TX cells; and it was transiently decreased following addition of IGF-1 to T98G TX cells for a limited time interval (**Fig 7** **B, C**). At greater than 120 min, its expression returned to a high level. The same result was obtained from experiments using HG-2 TX cells (data not shown). These data, therefore, demonstrate that expression of pStat1 and pStat3 was differentially regulated in Glioblastoma cancer cells in response to IGF-1 growth factor signaling, and, that pStat1 and pStat3 may have different roles in regulating expression of the TAP-1 gene.

## Discussion and Summary

Previous data showed that down-regulation in IGF-1 leads to an increase in cell surface MHC-1 [16]–[21], [25], [26]. This led to the hypothesis that decrease in intracellular IGF-1 would enhance components of the endogenous antigen processing and presentation pathway. The decrease in expression of endogenously processed tumor cell antigens in cancer tissues and cancer cell lines is a well-reported phenomenon [10]–[12], [27], [28]. It was previously demonstrated that the reverse of this process could be obtained by down-regulation in the expression of IL-10 [29]. We show in this paper an association between down–regulation in expression of IGF-1 and enhancement in the cell surface expression of HLA class 1 molecules. Along with this, there is a concomitant increase in the TAP-1, TAP-2, LMP-2 and LMP-7 components of the endogenous antigen presentation pathway.

Our previously reported work demonstrated enhancement in survival of animals that is consistent with immunity in four different animal model systems in which the intracellular expression of IGF-1 was down-regulated by transfection with vector expressing an IGF-1 antisense RNA or by transfection with vector expressing an IGF-1 RNA that can form a triple-helix oligonucleotide sequence with IGF-1 DNA [15]–[21]. The established role for the IGF-1 molecule in early differentiation of tissues as well as in cell proliferation, and, the possible need for the developing embryo to modulate the immune reaction toward protein antigens specifically expressed from the male parental genes provide a teleological rationale for a dual role in its regulation of development and immunity [30]–[32]. This together with the well reported anti- apoptotic effect of IGF-1 on programmed cell death provides insight into fundamental mechanisms for a causal role of this molecule in the progression toward frankly invasive cancer. One explanation for the results obtained, would concern whether the impact of IGF-1 is directed to selection of a specific subset of cells rather than to the modulation of IGF-1 in a given glial cell fraction. The care to select cloned cell fractions as starting material would seem to rule against this possibility. In addition, the reversal of the up-regulation in antigen processing machinery by addition of IGF-1 to culture medium would also tend to rule against this possibility. Furthermore, the morphological characteristics of transfected cells do not differ from the parental non-transfected cells. In addition, and importantly, similar results were obtained using the ATCC T98G stably cloned cell line of Glioblastoma as a standard control. Thus, we conclude that the decrease in the antigen processing machinery is affected by cell content of IGF-1.

Although a one base deletion of the TAP-1 promoter sequence of a melanoma cell line has been reported [33], other reports document that the decreased expression of TAP-1, 2 and LMP-2, 7 in cancer cell lines can be modulated or rescued by induction with IFN-γ [34]–[36]. Here we report that the deficiencies can be rescued by transfection of HGB cells with a vector expressing antisense IGF-1 RNA and/or by exogenous addition of antibody to IGF-1 receptor. We show further that the rescue can be aborted by addition of IGF-1 to culture medium (**Fig 7**).

The appropriate regulation of transport associated proteins and large multicatalytic proteasomes is critical for initiation and continuation of the cellular immune response through the endogenous antigen process pathway [28]. The TAP-1 and LMP-2, constituents of this processing pathway are interferon-gamma (IFN-γ) inducible genes. TAP-1 and LMP-2 were reported to be up-regulated or rescued by induction of IFN-γ via tyrosine phosphorylation of Stat 1 (signaling transducer and activator of transcription -1) [37]–[40]. We report in this paper that the restoration of TAP-1 and LMP-2 by down-regulation of IGF-1 in Glioblastoma cells was not related to the tyrosine phosphorylation of STAT 1, i.e. there was no pSTAT 1 detected in either wild type Glioblastoma cells or in cells transfected with the pAnti-IGF-1 vector that expresses IGF-1 antisense RNA and in which expression of TAP-1 and LMP-2 were restored by induction of the MT-1 promoter of pAnti IGF-1 in the absence of serum. There was also no pSTAT 1 detected in the pAnti IGF-1 transfected cells when IGF-1 was exogenously added to the serum-free culture medium (**Fig 7**). That is, the down-regulation of TAP-1 and LMP-2 in cells and/or the restoration of TAP1 by down-regulation of IGF-1 in these tumor cells are pSTAT 1 independent. Thus, we assume that the mechanism for the restoration of TAP-1 and LMP-2 by down-regulating IGF-1 is different, or partially different, from the one in which restoration of expression of genes by induction of IFN-γ occur in cancer cells. In the experiments described here, we found that the restoration of TAP-1 and LMP-2 may be related to the phosphorylation of STAT 3. Firstly, pSTAT 3 was detected in pAnti IGF-1 transfected, IGF-1 down-regulated T98G cells. Secondly, the exogenous addition of IGF-1 led to suppression in expression of pSTAT 3 for up to 6 hours; this suppression is paralleled by suppression in expression of TAP-1 (**Fig 7** **B, C**). These data show that STAT 3 may have a tumor-suppressive function in Glioblastoma cells, such as in the T98G cell line. This is similar to the findings of the unexpected Stat 3 function linked to PTEN gene activities in brain cancer cells by Bonni A, et al. [41]. Moreover, STAT 3 is an important transcription factor, and, activated STAT 3 can also bind to GAS element-like sequence or ISRE element to activate a promoter of downstream genes [42], [43]. Accordingly, we postulate, that STAT 3 may have a role in the restoration of TAP-1 and LMP-2 in IGF-1 down-regulated Glioblastoma cells. Further investigation is needed to elucidate the mechanisms involved in the modulation of antigen processing machinery by down-regulation of IGF-1 in cancer cells. **Fig 7** **B** also shows the effect of IGF-1 on expression of pAkt. PAkt was not detectable in pAnti IGF-1 transfected T98G cells cultured in serum-free medium plus 50 uM Zn2+. It was, however, detected 30–60 min after addition of IGF-1. This suggests that IGF-1 stimulates the PI3K/Akt signaling pathway, and is consistent with the work of others [44]. It is very likely that inhibition of IGF-1 leads to down-regulation in expression of the MHC-1 antigen processing [45].

It is clear, however, that IGF-1, in addition to its other functions, can modulate the endogenous antigen processing machinery and possibly the immune response as well as having its known role in modulating the process of apoptosis. Furthermore, in those cancers that over-express this molecule, strategies for treatment that modulate IGF-1 have promise for leading to efficacious immuno-gene therapy.

## References

[1] MonacoJJ (1995) Pathways for the processing and presentation of antigens to T cells. J Leukoc Biol 57: 543–547.772241210.1002/jlb.57.4.543

[2] HofmannM, NussbaumAK, EmmerichNP, StoltzeL, SchildH (2001) Mechanisms of MHC class I-restricted antigen presentation. Expert Opin Ther Targets 5: 379–393.1254027210.1517/14728222.5.3.379

[3] FlutterB, GaoB (2004) MHC Class I antigen presentation – recently trimmed and well presented. Cell Mol Immunol 1: 22–30.16212917

[4] GroettrupM, van den BroekM, SchwartzK, MacagnoA, KhanS, et al (2001) Structural plasticity of the proteasome and its function in antigen processing. Crit Rev Immunol 21: 339–358.11922078

[5] NiedermannG (2002) Immunological functions of the proteasome. Curr Top Microbiol Immunol 268: 91–136.1208301010.1007/978-3-642-59414-4_5

[6] Lankat-ButtgereitB, TampeR (1999) The transporter associated with antigen processing TAP: structure and function. FEBS Lett 464: 108–112.1061848710.1016/s0014-5793(99)01676-2

[7] AbeleR, TampeR (2006) Modulation of the antigen transport machinery TAP by friends and enemies. FEBS Lett 580: 1156–1163.1635966510.1016/j.febslet.2005.11.048

[8] CresswellP, BanggiaN, DickT, DiedrichG (1999) The nature of the MHC Class I peptide loading complex. Immunol Rev 172: 21–28.1063193410.1111/j.1600-065x.1999.tb01353.x

[9] RaghavanM, Del CidN, RizviMS, PetersRL (2008) MHC class 1 assembly: Out and about. Trends Immunology 29: 436–443.10.1016/j.it.2008.06.004PMC277444818675588

[10] SeligerB, MaeurerMJ, FerroneS (1997) TAP off – tumor on. Immunol Today 18: 292–299.919011610.1016/s0167-5699(97)01052-9

[11] Thor StraatenP, KirkinAF, SeremetT, ZeuthenJ (1997) Expression of transporter associated with antigen processing 1 and 2 (TAP ½) in malignant melanoma cell lines. Int J Cancer 70: 582–586.905275910.1002/(sici)1097-0215(19970304)70:5<582::aid-ijc15>3.0.co;2-f

[12] VitaleM, RezzaniR, RodellaL, ZauliG, GrigolatoP, et al (1998) HLA class 1 antigen and transporter associated with antigen processing (TAP 1 and TAP 2) down-regulation in high-grade primary breast carcinoma lesions. Cancer Res 58: 737–742.9485029

[13] AlyssaJ, FranceJ, SyMS, HardingCV (1998) Down-regulation of the transporter for antigen presentation, proteasome subunits, and class 1 major histocompatibility complex in tumor cell lines. Cancer Res 58: 3600–3667.9721876

[14] MurrayJL, HunsonJM, RossMI, ZhangHZ, IoannidesCG (2000) Reduced recognition of metastatic melanoma cells by autologous MART-1 specific CTL: relationship to TAP expression. J Immunother 23: 28–35.1068713510.1097/00002371-200001000-00005

[15] TrojanJ, JohnsonT, RudinS, IlanJ, TykocinskiM, et al (1993) Treatment and prevention of rat glioblastoma by immunogenic C6 cells expressing antisense insulin-like growth factor 1 RNA. Science 259: 94–97.841850210.1126/science.8418502

[16] TrojanJ, JohnsonTR, RudinSD, BlosseyBK, AnthonyDD, et al (1994) Gene therapy of murine teratocarcinoma: separate functions for insulin-like growth factors 1 and 2 in immunogenicity and differentiation. Proc Natl Acad Sci USA 91: 6088–6092.801612010.1073/pnas.91.13.6088PMC44143

[17] Upegui-GonzalezLC, LyA, DucHT, PanY, AnthonyD, et al (2001) IGF-1 triple helix strategy in hepatoma treatment. Hepatogastroenterology. 48: 660–666.11462897

[18] Lafarge-FrayssinetC, DueHT, FrayssinetC, SarasinA, AnthonyD, et al (1997) Antisense insulin-like growth factor 1 transferred into a rat hepotoma cell line inhibits tumorigenesis by modulating major histocompatibility complex 1 cell surface expression. Cancer Gene Ther 4: 276–285.9345599

[19] TrojanJ, DucHT, Upegui-GonzalezLC, GouY, AnthonyD, et al (1996) Presence of MHC-1 and B-7 molecules in rat and human glioma cells expressing antisense IGF-1 mRNA. Neurosci Lett 212: 9–12.882375010.1016/0304-3940(96)12770-1

[20] AnthonyDD, PanYX, WuSG, ShenF, GuoYJ (1998) Ex vivo and in vivo anti-sense RNA strategies for treatment of cancer in humans. Adv Exp Med Biol 451: 27–34.1002684610.1007/978-1-4615-5357-1_5

[21] LiuY, TrojanJ, HabibN, AnthonyDD, WuM, et al (2000) Enhancement of immunogenicity of tumor cells by co-transfection with gene encoding antisense insulin-like growth factor-1 and B7.1 molecules. Cancer Gene Ther 7: 456–465.1076635210.1038/sj.cgt.7700137

[22] PanYX, AnthonyDD (2000) IGF-1 antisense strategies for cancer treatment. Methods Mol Med 35: 189–204.2139080710.1385/1-59259-086-1:189

[23] YatesJL, WarrenN, SugdenB (1985) Stable replication of plasmids derived from Epstein-Barr virus in various mammalian cells. Nature 313 812–815.298322410.1038/313812a0

[24] TrojanJ, BlosseyB, JohnsonT, RudinS, TykocinskiM, et al (1992) Loss of tumorigenicity of rat glioblastoma directed by episome-based antisense cDNA transcription of insulin-like growth factor 1. Proc Natl Acad Sci U S A 89: 4874–4878.159458710.1073/pnas.89.11.4874PMC49190

[25] LYA, BouchaudC, HeninD, PanY, AnthonyD, et al (2000) Expression of insulin-like growth factor-1 in rat glioma cells is associated with change in both immunogenicity and apoptosis. Neurosci Lett 281: 13–16.1068640410.1016/s0304-3940(00)00758-8

[26] LyA, DucHT, KalamaridesM, FrancoisJC, AnthonyD, et al (2001) Human glioma cells transformed by IGF-1 triple helix technology show immune and apoptotic characteristics determining cell selection for gene therapy of glioblastoma. Mol Pathol 54: 230–239.1147713710.1136/mp.54.4.230PMC1187073

[27] KamarashevJ, FerroneS, BoniR, NestleFO, BurgG, et al (2001) TAP1 down-regulation in primary melanoma lesions: an independent marker of poor prognosis. Int J Cancer 95: 23–28.1124130610.1002/1097-0215(20010120)95:1<23::aid-ijc1004>3.0.co;2-4

[28] Lankat-ButtgereitB, TampeR (2002) The transporter associated with antigen processing: function and implications in human diseases. Physiol Rev 82: 187–204.1177361210.1152/physrev.00025.2001

[29] PeterssonM, CharoJ, Salazar-OnfrayF, NoffzG, MohauptM, et al (1998) Constitutive IL-10 production accounts for the high NK sensitivity, low MHC class 1 expression, and poor transporter associated with antigen processing (TAP)-1/2 function in the prototype NK target YAC-1. J Immunol 161: 2099–2105.9725200

[30] GibsonJM, AplinJD, WhiteA, WestwoodM (2001) Regulation of IGF bioavailability in pregnancy. Mol Hum Reprod 7: 79–87.1113436410.1093/molehr/7.1.79

[31] BaikI, DevitoWJ, BallenK, BeckerPS, OkuliczW, et al (2005) Association of fetal hormone levels with stem cell potential: evidence for early life roots of human cancer. Cancer Res 65: 358–363.15665314

[32] GustafssonC, MjosbergJ, MatussekA, GeffersR, MatthiesenL, et al (2008) Gene expression profiling of human decidual macrophages: evidence for immunosuppressive phenotype. PloS One 3: e2078.1844620810.1371/journal.pone.0002078PMC2323105

[33] SeligerB, RitzU, AbeleR, BockM, TampeR, et al (2001) Immune escape of melanoma: first evidence of structural alterations in two distinct components of the MHC class 1 antigen processing pathway. Cancer Res 61: 8647–8650.11751378

[34] GuoY, YangT, LiuX, LuS, WenJ, et al (2002) Cis elements for transporter associated with antigen-processing-2 transcription: two new promoters and an essential role of the IFN response factor binding element in IFN-gamma-mediated activation of the transcription initiator. Int Immunol 14: 189–200.1180973810.1093/intimm/14.2.189

[35] ProckoE, GaudetR (2009) Antigen processing and presentation: TAPing into ABC transporters. Curr Opin Immunol 21: 84–91.1926145610.1016/j.coi.2009.02.003

[36] MatsuiM, MachidaS, Itani-YohdaT, AkatsukaT (2002) Downregulation of the proteasome subunits, transporter, and antigen presentation in hepatocellular carcinoma, and their restoration by interferon-gamma. J Gastroenterol Hepatol 17: 897 .1216496610.1046/j.1440-1746.2002.02837.x

[37] CramerLA, NelsonSL, KlemszMJ (2000) Synergistic induction of the Tap-1 gene by IFN-gamma and lipopolysaccharide in macrophages is regulated by STAT1. J Immunol 165: 3190– 3197.1097583410.4049/jimmunol.165.6.3190

[38] Chatterjee-KishoreM, KishoreR, HicklinDJ, MarincolaFM, FerroneS (1998) 10.1074/jbc.273.26.161779632673

[39] Different requirements for signal transducer and activator of transcription 1α and interferon requlatory factor 1 in the regulation of low molecular mass polypeptide 2 and transporter associated with antigen processing 1 gene expression. J Biol Chem 273: 16177–16183.10.1074/jbc.273.26.161779632673

[40] BeckS, AbdullaS, AldertonRP, GlynneRJ, GutIG, et al (1996) Evolutionary dynamics of non-coding sequences within the class II region of the human MHC. J Mol Biol 255: 1–13.856885810.1006/jmbi.1996.0001

[41] BrucetM, MarquesL, SebastianC, LloberasJ, CeladaA (2004) Regulation of murine Tap 1 and Lmp 2 genes in macrophages by interferon gamma is mediated by STAT1 and IRF-1. Genes Immun 5: 26–35.1473514610.1038/sj.gene.6364035

[42] De La IglesiaN, KonopkaG, PuramSV, ChanJA, BachooRM, et al (2008) Identification of a PTEN-regulated STAT3 brain tumor suppressor pathway. Genes Dev 22: 449–462.1825875210.1101/gad.1606508PMC2238667

[43] LiP, HarrisD, LiuZ, LiuJ, KeatingM, et al (2010) Stat3 activates the receptor tyrosine kinase like orphan receptor-1 gene in chronic lymphocytic leukemia cells. PLoS One 5: e11859.2068660610.1371/journal.pone.0011859PMC2912280

[44] GiulianiC, SajiM, BucciI, FioreG, LiberatoreM, et al (2006) Transcriptional regulation of major histocompatibility complex class I gene by insulin and IGF-1 in FRTL-5 thyroid cells. J Endocrinol 189: 605–615.1673179110.1677/joe.1.06486

[45] MaX, BaiY (2012) IGF-1 activates the PI3K/AKT signaling pathway via upregulation of secretory clusterin. Mol Med Report 6: 1433–1437.10.3892/mmr.2012.111023027041

[46] InoueM, MimuraK, IzawaS, ShiraishiK, InoueA, atal (2012) Expression of MHC class 1 on breast cancer cells correlates inversely with HER2 expression. Oncoimmunology 1: 1104–1110.2317025810.4161/onci.21056PMC3494624

